# MicroRNA-27 Inhibits Autophagy and Promotes Proliferation of Multiple Myeloma Cells by Targeting the NEDD4/Notch1 Axis

This article has been retracted.

**DOI:** 10.3389/fonc.2020.571914

**Published:** 2020-11-11

**Authors:** Feifei Che, Jiao Chen, Chunqian Wan, Xiaobing Huang

**Affiliations:** Department of Hematology, Sichuan Academy of Medical Science & Sichuan People's Hospital, Chengdu, China

**Keywords:** miR-27, NEDD4, Notch1, autophagy, multiple myeloma, ubiquitination, invasion, proliferation

## Abstract

Multiple myeloma (MM) is a malignant tumor disease that seriously affects the health of patients. Previous studies have shown the crucial role of autophagy in the development of MM. Therefore, the study aimed to study the effect of miR-27 on autophagy in MM via NEDD4/Notch1 axis. RT-qPCR or western blot analysis was used to detect the expression of miR-27, NEDD4, and Notch1 in bone marrow tissues and CD138+ plasma cells of patients and MM cells. After gain- and loss-of-function assays in MM cells, proliferation and invasion were assessed by clone formation and Transwell assays. Meanwhile, expression of autophagy-related proteins was measured by western blot analysis, followed by evaluation of autophagosomes and autophagic flow. The targeting relationship was evaluated by luciferase reporter assay, whereas the binding of NEDD4 to Notch1 protein was analyzed by co-immunoprecipitation. The ubiquitination level of Notch1 protein was detected. A nude mouse tumor model was established to determine the role of miR-27 in MM *in vivo*. miR-27 and Notch1 upregulation and NEDD4 downregulation were observed in bone marrow tissues and CD138+ plasma cells of patients and MM cells. miR-27 negatively targeted NEDD4, while NEDD4 could specifically bind to Notch1 protein to increase Notch1 ubiquitin degradation in MM cells. miR-27 or Notch1 overexpression or NEDD4 silencing diminished autophagy but enhanced proliferation and invasion of MM cells. miR-27 upregulation promoted the formation of subcutaneous tumor in nude mice. Collectively, miR-27 elevated Notch1 expression by targeting NEDD4 and promoted the development of MM by inhibiting cell autophagy, which provides a new idea and basis for MM treatment.

## Introduction

Multiple myeloma (MM) is a B-cell malignancy, which accounts for 1% of all cancers and 10% of all hematological malignancies across the globe (1). The pathological characterization of MM is the infiltration of monoclonal plasma cells in bone marrow, monoclonal immunoglobulin secreted by MM cells which can be detected in the blood and urine samples (2). A higher incidence rate of myeloma has been reported in the elderly, which is more frequently diagnosed in individuals aged between 60 and 70 years. However, the incidence rate of myeloma has been gradually increasing among younger people (3). Although multiple therapeutic drugs, autologous stem cell transplantation, and detection methods have been discovered in recent years, the 5-year survival rate of patients affected by MM is still no more than 40% (4).

A wide array of studies have revealed cytogenetic and epigenetic changes in MM cells, which influence cellular proliferation, apoptosis, autophagy, and metastasis through different mechanisms, including the regulatory effects of microRNAs (miRNAs) on the progression of MM (5). miRNAs are small single-stranded RNAs (19–22 nucleotide in length), which participate in various malignant biological processes of MM (6). Different effects have been identified for specific miRNAs on MM cells, including pro-tumoral and antitumoral properties. For example, aberrantly high expression of miR-15a and miR-16 has been unveiled in MM, which contributes to accelerated proliferative potential of MM cells (7). Meanwhile, a tumor-suppressive miR-215-5p was also identified in MM, which leads to apoptotic potential of MM cells through downregulating the PI3K/AKT/mTOR signaling pathway (8).

It is interesting to note that miRNA-27a is frequently overexpressed in a plethora of human carcinomas, including myeloma, where high expression of miR-27 was observed to predict unsatisfactory prognosis and to augment progression of human MM (9). However, the specific mechanism underlying the effects of miR-27 on myeloma still remains unclear. miR-27a-5p and miR-27-3p are two isoforms of mature miR-27a. miR-27 has been delineated to exert oncogenic effects on various kinds of cancers, such as osteosarcoma (10), gastric cancer (11), and thyroid cancer (12). Ye et al. (10) have highlighted that increased expression of miR-27-3p enhances cell-cycle progression of osteosarcoma through targeting inhibitor of growth family member five. However, Jiang *et al*. have illuminated that miR-27b repressed proliferation and invasion of non-small cell lung cancer cells through targeting Sp1 transcription factor (13). Whether miR-27 accelerates or inhibits MM progression needs to be further elaborated. Notably, autophagy has been uncovered to play a pivotal role in MM through influencing chemoresistance (14). In the present study, we predicted that autophagy-related protein, the E3 ubiquitin ligase neural precursor cell-expressed developmentally downregulated protein 4 (NEDD4), can be modulated by miR-27 based on bioinformatics analysis. In addition, Notch1 has been observed to be overexpressed in MM tissues (15) and to facilitate proliferation of MM cells (16), which can be degraded by NEDD4 (17).

This current study is designed to investigate whether miR-27 affects MM progression *in vitro* and *in vivo* as well as the regulatory effects of miR-27 on the NEDD4/Notch1/autophagy axis.

## Materials and Methods

### Ethics Statement

The study was performed with the approval of the Ethics Committee of Sichuan Academy of Medical Science & Sichuan People's Hospital. The experiments were in compliance with the guidelines of the *Declaration of Helsinki* on human medical research. All patients or their family were informed of the research purposes and provided their written informed consent prior to enrollment. All animal experiments were conducted with ratification of the Animal Committee of Sichuan Academy of Medical Science & Sichuan People's Hospital and in strict accordance with the recommendations in the guidelines for the care and use of laboratory animals published by the National Institutes of Health. Extensive efforts were made to ensure minimal suffering of the included animals.

### Specimens and Cell Culture

A total of 72 MM patients [55 males and 17 females with a median age of 56 (39–76) years] and 72 healthy donors [50 males and 22 females with a median age of 59 (36–71) years] were selected from the department of hematology of Sichuan Academy of Medical Science & Sichuan People's Hospital from March 2014 to March 2016. All MM patients were diagnosed by histopathological examination and met the World Health Organization diagnostic criteria.

### Isolation of Human Bone Marrow Blood Mononuclear Cells and CD138+ Plasma Cells

Mononuclear cells from bone marrow blood were isolated by Ficoll–Hypaque density gradient centrifugation. In brief, about 5 mL bone marrow blood was drawn from MM patients and healthy donors using the posterior superior iliac spine or anterior superior iliac spine as the puncture point and then was anticoagulated with heparin sodium. The bone marrow blood was mixed with 1 × phosphate-buffered saline (PBS) at 1:5 ratio, then slowly added into 2 mL lymphocyte separation solution (Gibco, Carlsbad, California, USA) along the tube wall, followed by 20-min centrifugation at 2,500 rpm. The rain fog layer between the upper layer and the middle layer (mononuclear cells) was collected and put into 5 mL of 1 × PBS and centrifuged at 1,500 rpm for 10 min at room temperature. The cells were washed twice and counted.

CD138+ magnetic beads (NO.130-051-301, Miltenyi Biotech GmbH, Bergisch Gladbach, Germany) were utilized to separate CD138+ plasma cells according to the manufacturer's instructions. Specifically, every 1 × 10^7^ cells were resuspended with 40 μL Magnetic Cell Sorting (MACS) buffer and collected in a centrifuge tube. The cells were mixed with 20 μL CD138 magnetic beads and incubated at 4°C for 15 min. Cells were mixed with 2 mL MACS buffer and centrifuged at 300 g and 20°C for 10 min. After discarding the supernatant, 500 mL MACS buffer was added to resuspend the cells. Cells were sorted on a sorting column, and impurities and CD138- cells were washed out to obtain CD138+ plasma cells. The supernatant was discarded after a 5-min cell centrifugation at 1,500 rpm and room temperature. After cell counting, 10% dimethyl sulfoxide was added into cells and mixed well. The cells were stored at −80°C after gradient cooling at 4°C for 30 min and −20°C for 30 min for subsequent experiments. Bone marrow CD138+ plasma cells of MM patients were MM group, and bone marrow CD138+ plasma cells of healthy donors were normal plasma cell (NPC) group.

### Reverse-Transcription Quantitative Polymerase Chain Reaction (RT-qPCR)

The TRIzol (Invitrogen, Carlsbad, CA, USA) method was used to extract total RNA from bone marrow blood, tissues, and cells. The NanoDrop 2000 micro ultraviolet spectrophotometer (1011U, NanoDrop Technologies, Inc., Rockland, ME, USA) was used to detect the concentration and purity of the extracted total RNA. cDNA was generated from RNA according to the manuals of TaqMan MicroRNA Assays Reverse Transcription primer (4427975, Applied Biosystems, Carlsbad, CA, USA)/PrimeScript RT reagent Kit (RR047A, Takara, Tokyo, Japan). miR-27, NEDD4, and Notch1 primers were synthesized by Takara (Table 1). RT-qPCR was conducted with TaqMan Multiplex Real-Time Solution (4461882, Thermo Fisher Scientific Inc., Waltham, Massachusetts, USA) on ABI 7500 quantitative PCR instrument (7500, Applied Biosystems). The relative transcription level of the target gene was calculated using the relative quantitative method (2^−ΔΔCT^ method) (18) normalized to glyceraldehyde-3-phosphate dehydrogenase (GAPDH, for NEDD4 and Notch1) and U6 (for miR-27).

**Table 1:** RT-qPCR primer sequences.

**Gene**	**Sequence**
miR-27	F: 5′-CGCCTTGAATCGGTGACACTT-3′
	R: 5′-GGCAAGTGTCACCGATTCAAG-3′
NEDD4	F: 5′-GCATGTTTGCCATCCTCCCA-3′
	R: 5′-AGCCAGGCTTGCAAGAATTAG-3′
Notch1	F: 5′-CGCACAAGGTGTCTTCCAG-3′
	R: 5′-AGGATCAGTGGCGTCGTG-3′
U6	F: 5′-GCTTCGGCAGCACATATACTAT-3′
	R: 5′-CGCTTCACGAATTTGCGTGCAT-3′
GAPDH	F: 5′-TATGATGATATCAAGAGGGTAGT-3′
	R: 5′-TGTATCCAAACTCATTGTCATAC-3′

### Cell Transfection

Human MM cell lines (U266, LP1, KMS11, and H929; American Type Culture Collection, Rockville, Maryland, USA) and human bone marrow normal plasma cell lines (NPCs, Oulu Biotechnology, Wuhan, China) were cultured in Roswell Park Memorial Institute (RPMI)-1640 medium (Gibco) containing 10% fetal bovine serum (Gibco), 100 μg/mL streptomycin, and 100 U/mL penicillin at 37°C in a 5% CO_2_ incubator (Thermo Fisher Scientific Inc.). Cells at logarithmic phase were trypsinized and seeded in a 6-well plate at 1 × 10^5^ cells per well and incubated for 24 h. When cell confluence reached about 50%, MM cells were transiently transfected follow the protocols of Lipofectamine 2000 (Invitrogen) with mimic negative control (NC), miR-27 mimic, inhibitor NC, miR-27 inhibitor, mimic NC + overexpression (oe)-NC, mimic NC + oe-NEDD4, miR-27 mimic + oe-NC, miR-27 mimic + oe-NEDD4, oe-NC, oe-NEDD4, small interfering RNA (si)-NC (5′-AUUGUAUGCGAUCGCAGACUU-3′), si-NEDD4 (si1-NEDD4: 5′-UAGAGCCUGGCUGGGUUGUUU-3′, si2-NEDD4: 5′-UUCCAUGAAUCUAGAAGAACA-3′, and si3-NEDD4: 5′-UUCAAUUGCCAUCUGAAGUUUAUCC-3′), mimic NC + si-NC, miR-27 mimic + si-NC, miR-27 mimic + si-Notch1 (si1-Notch1: 5′-TGGCGGGAAGTGTGAAGCG-3′, si2-Notch1: 5′-GGTGTCTTCCAGATCCTGA-3′, and si3-Notch1: 5′-GGACCAACTGTGACATCAA-3′), Agomir NC + sh-NC, Agomir miR-27 + sh-NC, or Agomir miR-27 + sh-Notch1. Plasmids, mimic, inhibitor, and Agomir were all purchased and synthesized in Sino biological (Beijing, China).

### Western Blot Analysis

Tissues or cells was added with phenylmethylsulfonyl fluoride-contained Radio-Immunoprecipitation assay lysate (Beyotime Biotechnology, Shanghai, China) and lysed on ice for 10 min. After centrifugation at 14,000 rpm and 4°C, the supernatant was harvested. The bicinchoninic acid (Pierce, Rockford, IL, USA) method was used to estimate the protein concentration of the protein. After a 1-h blocking with 5% skimmed milk powder at room temperature, the membrane was probed with primary rabbit antibodies from Abcam (Cambridge, UK) against autophagy-related protein 5 (ATG5; 1:10,000) and Beclin1 (1:1,000) and primary rabbit antibodies from Sigma (St Louis, MO, USA) against P62 (1:3,000), Light Chain 3 (LC3; 2 μg/mL), NEDD4 (1:2,000), and Notch1 (1:10,000) at 4°C overnight. After washing with phosphate-buffered saline with Tween 20 (PBST) at room temperature, the membrane was re-probed for 1 h at room temperature with horseradish peroxidase-labeled rabbit Immunoglobulin G (IgG) secondary antibodies (1:1,000, Santa Cruz Biotechnology Inc., Santa Cruz, CA, USA) and washed with PBST three times for 5 min each time. In the electrogenerated chemiluminescence solution (Thermo Fisher Scientific Inc.), the color reaction was carried out at room temperature, and then the results were developed and fixed using Bio-Rad ChemiDoc™ imaging system. GAPDH (1:1,000, ab22555, Abcam) was used as internal reference, and the protein bands were analyzed with ImageJ 2× software. Each experiment was repeated at least three times.

### Observation of the Number of Autophagosomes

The 1 × 10^6^ cells in each group were obtained into a 2-mL Eppendorf tube and centrifuged at 1,200 rpm and room temperature for 10 min to form a clump of cells. Then, 2.5% glutaraldehyde was slowly added along the wall of the tube, and cells were fixed at 4°C for 12 h. After refixing in 1% OsO4 for 1 h at room temperature, cells were embedded after immersion in acetone dehydration, and 50-nm ultrathin sections were prepared on an ultramicrotome (LKB-3 microtome, Stockholm, Sweden). After staining with uranyl acetate and lead citrate, sections were observed and photographed under a transmission electron microscope (TEM, HT7700, Tokyo, Japan). Fields of view were randomly selected to photograph three times. By counting the number of autophagosomes in random field of view of different treatment groups, the autophagic activity of cells was quantitatively analyzed.

### Autophagy Detection

According to the Lipofectamine 2000 (Invitrogen) transfection instructions, monomeric red fluorescent protein (mRFP)–green fluorescent protein (GFP)–LC3 plasmid (Hanbio Biotechnology, China) was transiently transfected into H929 myeloma cells. After 48 h, 250 nm autophagy activator rapamycin (RAPA) or 1 μm autophagy inhibitor 3-methyladenine (3-MA) was added into cells for a 12-h incubation. After nucleus staining with 4′,6-diamidino-2-phenylindole (Sigma), the cells were observed and photographed under a laser confocal microscope (Zeiss LSM 710, ZEISS, Germany). The increase in GFP and RFP double-positive yellow dots indicated the early formation of autophagy, and the increase in GFP-negative and RFP-positive red dots represented the formation of autophagy lysosome. The autophagy flow was evaluated by the color change of mRFP/GFP.

### Colony Formation Assay

The MM cells in the logarithmic growth phase were detached with 0.25% trypsin and titrated gently to single cells. The number of living cells was counted, and the cell density was adjusted to 1 × 10^6^ cells/mL. Each group of cells was inoculated with 500 cells per well in a 24-well plate containing 1 mL culture medium pre-heated at 37°C and then placed at 37°C in a 5% CO_2_ incubator for 2–3 weeks. The medium was renewed every 2–3 times. When the visible colonies appeared in the dish, the culture was terminated. The MM cells were fixed with 5 mL of 4% paraformaldehyde for 15 min. MM cells was added with GIMSA (Invitrogen) and stained for 10–30 min. Imaging and cell counting were performed under an inverted microscope (Leica DMi8-M, Germany). The clone formation rate (%) = number of clones formed/number of cells inoculated × 100%.

### Transwell Assay

After 24 h of harvesting in serum-free medium, the MM cells were digested, suspended in serum-free medium Opti-MEMI (Invitrogen) containing 10 g/L bovine serum albumin (Sigma), with the cell density adjusted to 3 × 10^4^ cells/mL. In the experiment, a 24-well 8-μm Transwell chamber (Corning Inc., Corning, New York, USA) was used. Before the experiment, 50 μL Matrigel (Sigma) was spread in the chamber, with three chambers in each group and 100 μL of cell suspension per chamber. The lower chamber was added with 600 μL of 10% RPMI-1640 medium and cultured at 37°C and 5% CO_2_. After 48 h, the chamber was fixed with 4% paraformaldehyde for 30 min, then placed in 0.2% Triton X-100 (Sigma) solution for 15 min, and stained with 0.05% gentian violet for 5 min. The number of stained cells was counted under an inverted microscope (Leica DMi8-M, Germany). Five visual fields were randomly selected for counting. The experiment was repeated three times.

### Luciferase Reporter Assay

The binding site fragments between miR-27 and NEDD4 mRNA 3′-untranslated region (UTR) and mutant fragments were inserted into the luciferase reporter vector Pmir-GLO Dual-Luciferase miRNA Target Expression Vectors (Promega, Madison, WI, USA), namely, reporter plasmids NEDD4-wild type (WT) and NEDD4-mutant type (MUT). NEDD4 luciferase reporter plasmids were co-transfected with mimic NC and miR-27 mimic into 293T cells (Oulu Biotechnology). Luciferase reporter gene detection was performed using a dual-luciferase reporter gene analysis system (Promega). Renilla luciferase was used as an internal reference, and the activation degree of the target reporter gene was compared based on the ratio of the firefly luciferase activity to Renilla luciferase activity.

### Co-immunoprecipitation (Co-IP) Assay

The cells were harvested after 48 h of treatment. The cells were lysed on ice for 30 min by cell lysis buffer containing a protease inhibitor. The lysate was centrifuged at 4°C and 12,000 rpm for 30 min, followed by collection of the supernatant. One part of lysate was utilized as input and added with 2 μg anti-rabbit IgG (NC, Sigma), and the other part of lysate was added with 2 μg anti-rabbit NEDD4 antibody (Sigma), followed by overnight incubation at 4°C. The 10-μL protein A agarose beads were washed with lysis buffer for three times (centrifugation at 3,000 rpm for 3 min each time). The pre-treated 10-μL protein A agarose beads were added to the cell lysate undergoing overnight incubation with the antibody at 4°C and cultured for 3 h to couple the antibody with protein A agarose beads. After the immunoprecipitation reaction, the agarose beads were centrifuged at 4°C and 3,000 rpm for 3 min to the bottom of the tube. After discarding the supernatant, the agarose beads were washed three times with 1 mL lysis buffer. After estimation of the protein concentration, 15 μL of 2 × sodium dodecyl sulfate loading buffer was added into the cells and boiled for 5 min. Western blot analysis was performed.

### Determination of Protein Half-Lives

The cells transfected with the plasmid of interest for 24 h were evenly distributed in six cell culture dishes (6 cm). After 24 h, 200 μg/mL protein synthesis inhibitor [cycloheximide (CHX)] was added. Cells were collected at different time points (0, 2, 4, 6, 8, and 10 h). Western blot analysis was used to detect the expression of Notch1 (anti-Rabbit, Sigma).

### Protein Ubiquitination Analysis

MM cells were transfected with different plasmids. After 48 h, MM cells were added with 20 μmol/L protease inhibitor MG-132 and cultured for 6 h. Then, cell lysis buffer containing protease inhibitors was added into MM cells for 30-min lysing on ice. According to the method of Co-IP, Notch1 (anti-Rabbit, Sigma) was precipitated to obtain a protein immunoprecipitation complex. Western blot analysis was adopted to detect the expression of Notch1 (anti-Rabbit, Sigma) and Ubiquitin (anti-Rabbit, 1:10,000, Abcam).

### Xenograft in Nude Mouse Models

Thirty-six male Balb/c nude mice (aged 5 weeks, weighing 18–22 g) at specific pathogen-free grades were purchased from Shanghai Slac Experimental Animal Co., Ltd. (Shanghai China). Animals were housed in specific pathogen-free facilities and raised separately during the experiment. Suspension of MM cells (1 × 10^6^ cells/200 μL) transfected with Agomir NC + sh-NC, Agomir miR-27 + sh-NC, and Agomir miR-27 + sh-Notch1 were inoculated subcutaneously into the right hind leg of nude mice (*n* = 12/treatment). Tumor formation experiment lasted for 4 weeks. Then, we observed and measured the tumor size every 7 days in the same environment. The size of the tumor was calculated as the volume = (length × width)^2^/2. The mice were euthanized by cervical dislocation after 4 weeks of inoculation, and the tumor tissues were obtained, photographed, weighed, and measured.

### Statistical Analysis

Statistical analysis was performed using SPSS 21.0 (IBM Corp. Armonk, NY, USA). Measurement data were shown as mean ± standard deviation (SD). Unpaired *t*-test was employed to compare data between two groups. One-way analysis of variance (ANOVA) was applied for comparison among multiple groups, followed by Tukey's *post hoc* test. Tumor volume at different time points was compared using repeated-measures ANOVA, and other data at different time points were compared using two-way ANOVA. The Kaplan–Meier method was used to calculate the survival rate of patients. Pearson correlation analysis was adopted to observe the correlation of observed indicators. *p* < 0.05 was considered to be statistically significant.

## Results

### MiR-27 Is Highly Expressed in MM Tissues and Cells and Is Related to the Poor Prognosis of Patients

First, the expression of miR-27 in bone marrow of 72 MM patients (tumor group) and 72 healthy donors (normal group) was determined using RT-qPCR. The results indicated that the expression of miR-27 was significantly increased in bone marrow of MM patients compared to bone marrow of healthy donors (*p* < 0.05, Figure 1A). The patients were assigned into a high expression group and a low expression group according to the median expression of miR-27, and the Kaplan–Meier method was used to analyze the correlation between miR-27 expression and overall survival (OS) in patients with MM. The results demonstrated that the OS in the high expression group was significantly lower than that in the low expression group (Figure 1B). Mononuclear cells from bone marrow blood were isolated by Ficoll–Hypaque density gradient centrifugation, and CD138+ plasma cells were sorted by CD138+ magnetic beads. The expression of miR-27 was detected in bone marrow plasma cells of MM patients (MM group) and human normal bone marrow plasma cells (NPC group) by RT-qPCR, which showed that miR-27 expression was higher in bone marrow plasma cells of MM patients than in NPCs (*p* < 0.05, Figure 1C). Compared to NPCs, ATG5 and Beclin1 expression and LC3II/LC3I ratio were significantly decreased by the expression of P62 which was significantly increased in bone marrow CD138+ plasma cells of MM patients (*p* < 0.05, Figure 1D). These results suggested that the autophagy level in MM tumor cells was significantly lower than that of normal bone marrow plasma cells.

**Figure 1:** miR-27 is overexpressed in MM tissues and cells and is related to the poor prognosis of patients. **(A)**, miR-27 expression in bone marrow of MM patients (*n* = 72) and healthy donors (*n* = 72) detected by RT-qPCR. *p < 0.05 compared with bone marrow of healthy donors. **(B)**, The correlation between miR-27 expression and OS of the patient (*n* = 72) analyzed by Kaplan–Meier. **(C)**, The expression of miR-27 in bone marrow plasma cells from MM patients and NPCs detected by RT-qPCR (*n* = 72). *p < 0.05 compared with NPCs. **(D)**, Western blot analysis of the protein expression of autophagy-related proteins (ATG5, Beclin1, LC3 II/LC3 I, and P62) in bone marrow plasma cells from MM patients and NPCs. *p < 0.05 compared with NPCs. **(E)**, miR-27 expression in NPCs, U266, LP1, KMS11, and H929 detected by RT-qPCR. *p < 0.05 compared with NPCs. **(F)**, The protein expression of autophagy-related proteins (ATG5, Beclin1, LC3 II/LC3 I, and P62) in H929 cells and NPCs detected by western blot analysis. *p < 0.05 compared with NPCs. The data were measurement data and expressed as mean ± standard deviation. Unpaired *t*-test was used for comparison between two groups, and one-way ANOVA was used for comparison among multiple groups. The cell experiment was repeated three times.

In order to screen the cell lines for subsequent experiments, we detected the expression of miR-27 in four MM cell lines (U266, LP1, KMS11, and H9294) and NPCs by RT-qPCR. The results demonstrated that the expression of miR-27 was significantly higher in four MM cell lines than in NPCs, especially in H929 cell lines (*p* < 0.05). Therefore, the follow-up experiments were conducted on H929 cell lines (Figure 1E). Compared with NPCs, ATG5 and Beclin1 expression and LC3II/LC3I ratio were remarkably decreased in H929 cells and the expression of P62 was significantly increased (Figure 1F). The above results indicated that miR-27 was highly expressed in MM tissues and cell lines, which was correlated with the poor prognosis of MM patients and the deceased autophagy in MM cells.

### MiR-27 Inhibits Autophagy to Promote the Proliferation and Invasion of MM Cells

To investigate the function of miR-27 in autophagy, proliferation, and invasion, H929 cells were treated with miR-27 mimic and RAPA. After transfection with miR-27 mimic or miR-27 mimic + RAPA, the expression of miR-27 was significantly increased in H929 compared with mimic NC treatment (*p* < 0.05, Figure 2A). The H929 cells were further treated with miR-27 inhibitor and autophagy inhibitor 3-MA for detection. Compared with H929 cells treated with inhibitor-NC, miR-27 expression was potently diminished in H929 cells treated with miR-27 inhibitor or miR-27 inhibitor + 3-MA (*p* < 0.05, Figure 2B). As revealed in Figures 2C,D, the number of autophagosomes and autophagic flow were reduced in H929 cells by miR-27 mimic, which was annulled by RAPA treatment. However, the miR-27 inhibitor decreased the number of autophagosomes and autophagic flow in H929 cells, and additional treatment with 3-MA abrogated these trends. Colony formation and Transwell assays displayed that H929 cell proliferation and invasion were accelerated by treatment with the miR-27 mimic, which was neutralized by additional RAPA treatment. Moreover, H929 cell proliferation and invasion were reduced in response to the miR-27 inhibitor, which was normalized by treatment with 3-MA (*p* < 0.05, Figures 2E,F). In summary, miR-27 overexpression inhibited autophagy and then promoted the proliferation and invasion of MM cells.

**Figure 2:** miR-27 represses autophagy and promotes the proliferation and invasion of MM cells. **(A)**, miR-27 expression in H929 cells transfected with mimic NC, miR-27 mimic, and miR-27 mimic + RAPA detected by RT-qPCR. *p < 0.05 compared with H929 cells transfected with mimic NC; ns means no significant difference. **(B)**, miR-27 expression in H929 cells transfected with inhibitor NC, miR-27 inhibitor, or miR-27 inhibitor + 3-MA detected by RT-qPCR. *p < 0.05 compared with H929 cells transfected with inhibitor NC; ns means no significant difference. H929 cells were transfected with mimic NC, miR-27 mimic, miR-27 mimic + RAPA, inhibitor NC, miR-27 inhibitor, or miR-27 inhibitor + 3-MA. **(C)**, The number of autophagosome in H929 cells detected by TEM (bar = 1 μm). **(D)**, Autophagic flow in H929 cells (bar = 25 μm). **(E)**, Proliferative capacity of H929 cells detected by clone formation assay. **(F)**, Invasion ability of H929 cells determined by Transwell assay (bar = 50 μm) *p < 0.05 compared with H929 cells transfected with mimic NC or inhibitor NC. The data were measurement data and expressed as mean ± standard deviation. Unpaired *t*-test was used for comparison between two groups, and one-way ANOVA was used for comparison among multiple groups. The cell experiment was repeated three times.

### MiR-27 Targets and Inhibits E3 Ubiquitin Ligase NEDD4 in MM Cells

In order to further explore the mechanism of miR-27 in MM, we conducted bioinformatics analysis of the predicted targets of miR-27, which predicted binding sites and targeted the relationship between miR-27 and NEDD4 (Figure 3A). To further investigate whether miR-27 affects autophagy of MM cells by regulating NEDD4 expression, NEDD4 expression was determined in the bone marrow of MM patients and healthy donors by RT-qPCR. The results found that NEDD4 expression was significantly reduced in the bone marrow of MM patients in contrast to bone marrow of healthy donors (*p* < 0.05, Figure 3B), contrary to miR-27 expression (Figure 3C). According to the median expression of NEDD4, the patients were assigned into a NEDD4 high expression group and a NEDD4 low expression group. Then, Kaplan–Meier analysis results showed that patients with low NEDD4 expression had lower OS than the patients with high NEDD4 expression (Figure 3D). Then, NEDD4 expression was measured in bone marrow CD138+ plasma cells of MM patients and NPCs. The results showed that both mRNA and protein levels of NEDD4 were significantly reduced in bone marrow CD138+ plasma cells of MM patients in comparison to NPCs (*p* < 0.05, Figures 3E,F). From the results above, we speculate that miR-27 may play a role in MM by regulating NEDD4.

**Figure 3:** miR-27 negatively targets ubiquitin ligase NEDD4 in MM cells. **(A)**, Bioinformatics analysis predicted the targeting relationship and binding sites between miR-27 and NEDD4. **(B)**, NEDD4 expression in bone marrow of MM patients (*n* = 72) and healthy donors (*n* = 72) detected by RT-qPCR. *p < 0.05 compared with bone marrow of healthy donors. **(C)**, Correlation analysis between miR-27 and NEDD4 expression in bone marrow of MM patients (*n* = 72) and healthy donors (*n* = 72). **(D)**, Correlation of NEDD4 expression with OS of patients analyzed by Kaplan–Meier. **(E)**, The expression of NEDD4 mRNA in bone marrow plasma cells from MM patients and NPCs detected by RT-qPCR. **(F)**, The expression of NEDD4 protein in bone marrow plasma cells from MM patients and NPCs detected by western blot analysis. N, NPC cell; M, MM cell. *p < 0.05 compared with NPCs. **(G)**, Luciferase report to show the targeting relationship between miR-27 and NEDD4 mRNA. *p < 0.05 compared with mimic NC treatment. **(H)**, Expression of NEDD4 mRNA in H929 cells treated with mimic NC or miR-27 mimic detected by RT-qPCR. **(I)**, Expression of NEDD4 protein in H929 cells treated with mimic NC or miR-27 mimic detected by western blot analysis. *p < 0.05 compared with H929 cells treated with mimic NC. **(J)**, Expression of NEDD4 mRNA in H929 cells treated with inhibitor NC or miR-27 inhibitor detected by RT-qPCR. **(K)**, Expression of NEDD4 protein in H929 cells treated with inhibitor NC or miR-27 inhibitor detected by western blot analysis. *p < 0.05 compared with H929 cells treated with inhibitor NC. The data were measurement data and expressed as mean ± standard deviation. Unpaired *t*-test was used for comparison between two groups. Pearson correlation analysis was used to analyze the relationship between miR-27 and NEDD4 expression. The Kaplan–Meier method was used to analyze the correlation between NEDD4 expression and OS in patients. The cell experiment was repeated three times.

Luciferase results depicted that the luciferase activity of the NEDD4-WT plasmid was lowered by miR-27 mimic (*p* < 0.05), and the luciferase activity of the NEDD4-MUT plasmid did not change (Figure 3G), which indicated that NEDD4 could bind to miR-27. RT-qPCR and western blot analysis described that expression of NEDD4 was strikingly diminished by miR-27 mimic (*p* < 0.05, Figures 3H,I) but was enhanced by miR-27 inhibitor (*p* < 0.05, Figures 3J,K). The results suggested that miR-27 could target E3 ubiquitin ligase NEDD4 in MM cells.

### NEDD4 Overexpression Reverses the Role of miR-27 to Promote Autophagy and Inhibit Proliferation and Invasion of MM Cells

In order to verify whether miR-27 affects MM cell autophagy by targeting NEDD4, H929 cells were transfected with mimic NC + oe-NC, mimic NC + oe-NEDD4, miR-27 mimic + oe-NC, or miR-27 mimic + oe-NEDD4. Next, miR-27 expression was detected by RT-qPCR (Figure 4A), and NEDD4 expression was measured by RT-qPCR and western blot analysis (Figures 4B,C). miR-27 expression was augmented, but NEDD4 expression was decreased in miR-27 mimic-transfected H929 cells. However, miR-27 expression was unchanged and NEDD4 expression was increased in NEDD4-overexpressed H929 cells. In addition, compared to the treatment with miR-27 mimic + oe-NC, treatment with miR-27 mimic + oe-NEDD4 did not affect miR-27 expression but elevated NEDD4 expression. As documented in Figures 4D,E, the number of autophagosomes and autophagic flow in H929 cells were lowered by miR-27 mimic but enhanced by oe-NEDD4, which was neutralized by treatment with miR-27 mimic + oe-NEDD4. Based on results of colony formation (Figure 4F) and Transwell (Figure 4G) assays, miR-27 mimic augmented but oe-NEDD4 diminished H929 cell proliferation and invasion. Moreover, in the presence of miR-27 mimic, NEDD4 overexpression caused a decline in H929 cell proliferation and invasion. Collectively, NEDD4 overexpression inhibited the effects of miR-27 on MM by promoting cell autophagy but repressing cell proliferation and invasion.

**Figure 4:** NEDD4 negates the role of miR-27 on autophagy, proliferation, and invasion of MM cells. H929 cells were transfected with mimic NC + oe-NC, mimic NC + oe-NEDD4, miR-27 mimic + oe-NC, or miR-27 mimic + oe-NEDD4. **(A)**, The expression of miR-27 in H929 cells measured by RT-qPCR. **(B)**, The expression of NEDD4 in H929 cells detected by RT-Qpcr. **(C)**, The expression of NEDD4 and autophagy-related proteins (ATG5, Beclin1, LC3 II/LC3 I, and P62) detected by western blot analysis. **(D)**, The number of autophagosomes in H929 cells detected by TEM (bar = 1 μm). **(E)**, Autophagic flow in H929 cells (bar = 25 μm). **(F)**, Proliferation ability of H929 cells measured by colon formation assay. **(G)**, Invasion ability of H929 cells assessed by Transwell assay (bar = 50 μm). *p < 0.05 compared with H929 cells transfected with mimic NC + oe-NC, ^#^*p* < 0.05 compared with H929 cells transfected with miR-27 mimic + oe-NC. The data were measurement data and expressed as mean ± standard deviation. One-way ANOVA was used for comparison among multiple groups. The cell experiment was repeated three times.

### NEDD4 Binds Specifically to Notch1 Protein and Increases Notch1 Ubiquitination and Degradation in MM Cells

Next, we explored whether NEDD4 plays a pivotal role in MM development via Notch1. Notch1 expression was evaluated in bone marrow of MM patients and healthy donors using RT-qPCR, which demonstrated an appreciably higher Notch1 expression in the bone marrow of MM patients than in the bone marrow of healthy donors (*p* < 0.05, Figure 5A), which was inversely correlated with NEDD4 expression (Figure 5B). Compared with NPCs, Notch1 expression was significantly increased at both mRNA and protein levels in bone marrow CD138+ plasma cells of MM patients (*p* < 0.05, Figures 5C,D). After NEDD4 was overexpressed in H929 cells, RT-qPCR and western blot analysis results showed that NEDD4 expression was prominently enhanced, but Notch1 protein level was decreased significantly along with unchanged mRNA level of Notch1 (*p* < 0.05, Figures 5E,F). Therefore, we speculate that NEDD4, as an E3 enzyme, might degrade the Notch1 protein.

**Figure 5:** NEDD4 specifically binds to Notch1 protein and mediate the ubiquitination and degradation of Notch1 protein in MM cells. **(A)**, Expression of Notch1 in bone marrow of MM patients (*n* = 72) and healthy donors (*n* = 72) detected by RT-qPCR. *p < 0.05 compared with bone marrow of healthy donors. **(B)**, Correlation analysis between NEDD4 and Notch1 expression in bone marrow of MM patients (*n* = 72) and healthy donors (*n* = 72). **(C)**, The expression of Notch1 mRNA in bone marrow plasma cells from MM patients and NPCs detected by RT-qPCR. **(D)**, The expression of Notch1 protein in bone marrow plasma cells from MM patients and NPCs detected by western blot analysis. N, NPC cell; M, MM cell. *p < 0.05 compared with NPCs. **(E)**, Expression of NEDD4 and Notch1 in H929 cells transfected with oe-NC or oe-NEDD4 detected by RT-qPCR. **(F)**, Expression of NEDD4 and Notch1 in H929 cells transfected with oe-NC or oe-NEDD4 detected by western blot analysis. *p < 0.05 compared with H929 cells transfected with oe-NC. **(G)**, Co-IP result of binding between NEDD4 and Notch1 in H929 cells transfected with oe-NC or oe-NEDD4. **(H)**, Expression of NEDD4 and Notch1 mRNA in H929 cells transfected with si-NC, si1-NEDD4, si2-NEDD4, or si3-NEDD4 detected by RT-qPCR. **(I)**, Expression of NEDD4 and Notch1 protein in H929 cells transfected with si-NC, si1-NEDD4, si2-NEDD4, and si3-NEDD4 detected by western blot analysis. *p < 0.05 compared with H929 cells transfected with si-NC. **(J)**, Co-IP result of binding between NEDD4 and Notch1 in H929 cells transfected with si-NC or si-NEDD4. **(K)**, The ubiquitination level of Notch1 in H929 cells after treatment with oe-NEDD4 and MG-132. *p < 0.05 compared with H929 cells transfected with oe-NC, ^#^*p* < 0.05 compared with H929 cells treated with oe-NC + MG-132, ^&^*p* < 0.05 compared with H929 cells treated with oe-NEDD4. **(L)**, The ubiquitination level of Notch1 in H929 cells after silencing NEDD4. *p < 0.05 compared with H929 cells treated with si-NC. **(M)**, Half-life of Notch1 in H929 cells after overexpressing NEDD4. *p < 0.05 compared with H929 cells transfected with oe-NC. **(N)**, Half-life of Notch1 in H929 cells after silencing NEDD4. *p < 0.05 compared with H929 cells treated with si-NC. The result data were measurement data and expressed as mean ± standard deviation. Unpaired *t*-test was used for comparison between two groups, and one-way ANOVA was used for comparison among multiple groups. Pearson correlation was used to analyze the relationship between NEDD4 and Notch1, and data at different time points were compared using two-way analysis of variance. The cell experiment was repeated three times.

After overexpression of NEDD4 in H929 cells, the co-immunoprecipitation experiment revealed that the amount of Notch1 protein bound by NEDD4 protein was significantly increased (Figure 5G). Meanwhile, the ubiquitination level of Notch1 protein was also increased, but Notch1 protein expression was decreased by overexpressing NEDD4 in H929 cells, which was reversed by additional treatment with ubiquitination degradation inhibitor MG-132 (*p* < 0.05, Figure 5K). Further, the protein half-life of Notch1 was examined, and it was manifested that the half-life of Notch1 protein was shortened after overexpression of NEDD4 in H929 cells (Figure 5M). The above results demonstrated that the overexpression of NEDD4 in H929 cells reduced the stability of Notch1 and accelerated its ubiquitination and degradation.

In addition, H929 cells were transfected with three siRNAs targeting NEDD4 to silence NEDD4. As a result, compared with si-NC treatment, NEDD4 expression was severely reduced after transfection with siRNAs targeting NEDD4 (*p* < 0.05). si1-NEDD4 had the highest silencing efficiency of NEDD4, so this sequence was used for subsequent experiments (Figures 5H,I). After silencing NEDD4 in H929 cells, the expression of Notch1 was significantly increased (*p* < 0.05, Figures 5H,I); the amount of Notch1 protein bound by NEDD4 protein was markedly reduced (Figure 5J), the ubiquitination level of Notch1 protein decreased significantly (Figure 5L) and the half-life of Notch1 protein increased (Figure 5N). In summary, it was shown that in MM cells, NEDD4 could specifically bind to Notch1 protein and promote the ubiquitination and degradation of Notch1 protein.

### MiR-27 Inhibits Cellular Autophagy by Targeting NEDD4 and Upregulating Notch1 to Promote the Development of MM

In order to verify whether miR-27 regulates the level of autophagy through the NEDD4/Notch1 axis and thus affects the development of MM, H929 cells were transfected with 3 siRNAs targeting Notch1 to silence Notch1. Both the mRNA and protein levels of Notch1 were significantly reduced in response to 3 siRNAs targeting Notch1 compared to si-NC treatment (*p* < 0.05). si1-Notch1 was used for subsequent experiments because it had the highest silencing efficiency (Figures 6A,B). Then, H929 cells were transfected with mimic NC + si-NC, miR-27 mimic + si-NC, or miR-27 mimic + si-Notch1. When miR-27 mimic was transfected into H929 cells, the autophagy was noticeably reduced, and proliferation and invasion ability were increased significantly. In the presence of miR-27 mimic, si-Notch1 did not change miR-27 and NEDD4 expression but diminished both the mRNA and protein levels of Notch1 (Figures 6C–E). Furthermore, the number of autophagosomes and autophagic flow were increased observably, but the proliferation and invasion were reduced substantially by silencing Notch1 in the presence of miR-27 mimic (*p* < 0.05, Figures 6F–I).

**Figure 6:** miR-27 suppresses autophagy by inhibiting NEDD4 and activating Notch1 to promote the development of MM. **(A)**, Notch1 expression detected by RT-qPCR in H929 cells transfected with si-NC, si1-Notch1, si2-Notch1, or si3-Notch1. **(B)**, Notch1 expression detected by western blot analysis in H929 cells transfected with si-NC, si1-Notch1, si2-Notch1, and si3-Notch1. *p < 0.05 compared with H929 cells transfected with si-NC. H929 cells were transfected with mimic NC + si-NC, miR-27 mimic + si-NC, or miR-27 mimic + si-Notch1. **(C)**, miR-27 expression in H929 cells detected by RT-qPCR. **(D)**, NEDD4 and Notch1 mRNA expression in H929 cells detected by RT-qPCR **(E)**, NEDD4 and Notch1 protein expression in H929 cells detected by western blot analysis. **(F)**, The number of autophagosomes in H929 cells (bar = 1 μm). **(G)**, Autophagic flow in H929 cells (bar = 25 μm). **(H)**, H929 cell proliferation detected by colon formation assay. **(I)**, The invasion ability of H929 cells assessed by Transwell assay (bar = 50 μm) *p < 0.05 compared with H929 cells transfected with mimic NC + si-NC, ^#^*p* < 0.05 compared with H929 cells transfected with miR-27 mimic + si-NC. H929 cells transfected with Agomir NC + sh-NC, Agomir miR-27 + sh-NC, or Agomir miR-27 + sh-Notch1 were subcutaneously injected into nude mice. **(J)**, Tumor volume of nude mice measured every 7 weeks (*n* = 12). **(K)**, The change in the trend of tumor size in mice within 4 weeks of inoculation of H929 cells (*n* = 12). **(L)**, Tumor weight of nude mice after 4 weeks of inoculation of H929 cells (*n* = 12). **(M)**, Expression of miR-27 in tumors detected by RT-qPCR. **(N)**, The expression of NEDD4 and Notch1 mRNA in the tumors detected by RT-qPCR. **(O)**, The expression of NEDD4 and Notch1 protein in the tumors detected by western blot analysis. *p < 0.05 compared with mice treated with Agomir NC + sh-NC, ^#^*p* < 0.05 compared with mice treated with Agomir miR-27 + sh-NC. The data were measurement data and expressed as mean ± standard deviation. Repeated-measures ANOVA was used for comparison of the weight of tumors at different time points, and one-way ANOVA was used for comparison among multiple groups. The cell experiment was repeated three times.

To investigate the effect of miR-27 *in vivo*, H929 cells transfected with Agomir NC + sh-NC, Agomir miR-27 + sh-NC, or Agomir miR-27 + sh-Notch1 were subcutaneously injected into nude mice. The results showed that Agomir miR-27 significantly increased the tumorigenic ability of nude mice (Figures 6J–L), elevated the miR-27 expression (Figure 6M), reduced the mRNA and protein levels of NEDD4 (*p* < 0.05), and enhanced the Notch1 protein level with the mRNA expression of Notch1 unchanged, which was abrogated by silencing Notch1 except for the unchanged miR-27 and NEDD4 expression (*p* < 0.05, Figures 6N,O). The results above indicated that miR-27 inhibited cell autophagy by targeting NEDD4 and upregulating Notch1, thereby promoting the development of MM.

## Discussion

In this work, we delineated that miR-27 accelerated the proliferation and invasion of MM cells *in vitro* and in animal models through regulating the NEDD4/Notch1/autophagy axis. Furthermore, miR-27 and NEDD4 presented with the potential values of serving as prognostic markers in MM.

miR-27 has been reported to be associated with the prognosis of a variety of cancers, including MM, but little is known about its role in MM cell proliferation and invasion. In this study, we revealed that miR-27 was highly expressed in bone marrow tissues and CD138+ plasma cells of patients and MM cells and related to the poor prognosis of patients. Therefore, miR-27 exerted oncogenic effects on MM cells, which was consistent with many other researches. Mozos et al. (19) have suggested that miR-27 was upregulated in invasive endometrioid endometrial adenocarcinoma, and its expression was positively correlated with clinical staging. Accumulating evidence has indicated that miR-27 modulates apoptosis of cancer cells. Liu et al. (20) delineated that miR-27b restricted chemoresistance of oral squamous cell carcinoma to cisplatin and reduced the proliferative ability of cancer cells through downregulating the expression of Frizzled-7 and β-catenin. This corroborates the findings of this study, which demonstrated that miR-27 can inhibit autophagy and augment the proliferation and invasion potential of MM cells. In future studies, we will further study the effects of miR-27 on apoptosis and chemoresistance of MM cells *in vitro* and in animal models. It is also important for us to evaluate whether the serum expression of miR-27 is higher in MM patients, which enables miR-27 to be a potential serum detection indicator in MM patients in the future.

Further mechanistic exploration indicated that miR-27 inhibited the expression of E3 ubiquitin ligase NEDD4 in MM cells. In this work, we explained that miR-27 restricted the autophagy and enhanced the progression of MM through the NEDD4/Notch1 axis. NEDD4 could reverse the effectiveness of miR-27 and promote autophagy, thereby inhibiting the proliferation and invasion of myeloma cells. These findings support the oncogenic effects of miR-27, the involved mechanism of autophagy in MM pathogenesis, and the potential therapeutic values of targeting autophagy-related molecules in MM. For instance, Xu et al. (21) have indicated that miR-221/222 levels were increased in serum of patients with MM and their expression was positively correlated with dexamethasone sensitivity in MM cell lines. Autophagy can not only affect the survival of cancer cells but also participate in the mechanism for cell death and drug resistance. Moreover, miR-221/222 restricted cell autophagy through directly targeting ATG12 and p27^kip^ expression, which induced dexamethasone resistance in MM.

In this study, we further proceeded to clarify the regulatory mechanism of miR-27 through targeting the NEDD4/Notch1 axis in MM cells. It is noted that E3 ubiquitin ligase NEDD4 downregulation has been associated with unfavorable prognosis of MM patients, due to the contribution to drug resistance (22). Emerging studies documented that NEDD4 exerted a promotive regulation of autophagy through different mechanisms in different types of cells. Xie et al. (23) reported that NEDD4 was a positive regulator of autophagy through reducing the K48-mediated ubiquitination of PIK3C3 through recruiting USP13. In addition, another study has indicated that NEDD4 expedited cellular proliferation, metastatic ability, and induced autophagy in prostate carcinoma cells, which was associated with inhibition of the mTOR signaling pathway (24). The experimental data suggested that miR-27-mediated NEDD4 inhibition suppressed autophagy, proliferation, and metastasis of MM cells, which was implicated in the upregulation of Notch1. Specifically, NEDD4 can specifically bind to Notch1 protein and mediate the ubiquitination and degradation of Notch1 protein in MM cells. Prior evidence has identified upregulation of Notch1 in MM patients, which holds prognostic significance in the treatment of MM (25). Additionally, a previous immunohistochemical investigation by Skrtic et al. (26) has also proposed the implication of the Notch signaling behind the pathogenesis of MM.

## Conclusions

In summary, this study reported a regulatory mechanism targeting the miR-27/NEDD4/Notch1 axis in MM. The obtained findings define a potential role of miR-27 downregulation as a therapeutic target in MM. In future work, we will further investigate the effects of autophagy in MM treatment and conduct more researches to evaluate the clinical translation of pertinent molecules involved in the miR-27/NEDD4/Notch1/autophagy axis.

## Data Availability Statement

The original contributions presented in the study are included in the article/Supplementary Material, further inquiries can be directed to the corresponding author.

## Ethics Statement

The studies involving human participants were reviewed and approved by the Medical Ethics Committee of Sichuan Academy of Medical Science and Sichuan People's Hospital. The patients/participants provided their written informed consent to participate in this study. The animal study was reviewed and approved by the Animal Committee of Sichuan Academy of Medical Science and Sichuan People's Hospital.

## Author Contributions

FC and JC designed the study. CW and XH collated the data. FC, JC, and CW carried out data analyses. FC, JC, and XH produced the initial draft of the manuscript. All authors have read and approved the final submitted manuscript.

## Conflict of Interest

The authors declare that the research was conducted in the absence of any commercial or financial relationships that could be construed as a potential conflict of interest.
